# Theaflavin Chemistry and Its Health Benefits

This article has been retracted.

**DOI:** 10.1155/2021/6256618

**Published:** 2021-11-18

**Authors:** Zhiguo Shan, Muhammad Farrukh Nisar, Mingxi Li, Chunhua Zhang, Chunpeng (Craig) Wan

**Affiliations:** ^1^College of Agriculture and Forestry, Pu'er University, Pu'er 665099, China; ^2^Jiangxi Key Laboratory for Postharvest Technology and Nondestructive Testing of Fruits & Vegetables, College of Agronomy, Jiangxi Agricultural University, Nanchang 330045, China; ^3^Department of Physiology and Biochemistry, Cholistan University of Veterinary and Animal Sciences (CUVAS), Bahawalpur 63100, Pakistan; ^4^Research Center of Tea and Tea Culture, College of Agronomy, Jiangxi Agricultural University, Nanchang, Jiangxi, China

## Abstract

Huge epidemiological and clinical studies have confirmed that black tea is a rich source of health-promoting ingredients, such as catechins and theaflavins (TFs). Furthermore, TF derivatives mainly include theaflavin (TF1), theaflavin-3-gallate (TF2A), theaflavin-3′-gallate (TF2B), and theaflavin-3,3′-digallate (TF3). All of these TFs exhibit extensive usages in pharmaceutics, foods, and traditional medication systems. Various indepth studies reported that how TFs modulates health effects in cellular and molecular mechanisms. The available literature regarding the pharmacological activities of TFs has revealed that TF3 has remarkable anti-inflammatory, antioxidant, anticancer, antiobesity, antiosteoporotic, and antimicrobial properties, thus posing significant effects on human health. The current manuscript summarizes both the chemistry and various pharmacological effects of TFs on human health, lifestyle or aging associated diseases, and populations of gut microbiota. Furthermore, the biological potential of TFs has also been focused to provide a deeper understanding of its mechanism of action.

## 1. Introduction

Tea, is a dried leaf–infused beverage obtained from the leaves of a small shrub originally from China, has become the world's second popular beverage after water. Over 3 billion cups are being consumed every day worldwide [1, 2]. The major tea-exporting countries in 2017 are China (USD 1.6 billion), Sri Lanka (USD 1.5 billion), and Kenya (USD 1.4 billion), while the largest importing countries were Pakistan (USD 550 million), Russia (USD 525 million), and the United States (USD 487 million) [3]. A significant quantity of tea is also consumed in China main lands. For instance, the amount of tea consumed in China, India ,and Turkey during 2015 was more than in all other tea-consuming nations [4]. Over fifty countries are growing tea worldwide for its domestic usage as well as export product and hence employed almost 13 million people. A huge number of bioactive compounds have been identified in tea samples especially the polyphenols, flavonoids, and tannins. For instance, black tea have 30-40% polyphenols comprising mainly TFs, thearubigins (TRs), and bisflavonols [5].

Theaflavins (TFs) comprised of a large group of polyphenols abundantly present in black and oolong teas. TFs are the biflavonoid class consisting of a benzotropolone skeleton and accounting for about 2% of dried tea leaves. TFs are the main oxidation products of catechins and aggregates during the fermentation steps [5, 6]. TFs are formed by the oxidation of selected catechins (epicatechin and epigallocatechin-3-gallate) in presence of polyphenol oxidase and peroxidase enzymes [7]. During fermentation, the catechins get converted to TFs primarily the theaflavin (TF1), theaflavin-3-gallate (TF2A), theaflavin-3′-gallate (TF2B), theaflavin-3,3′-digallate (TF3) (Figure 1), and certain polymers of the arubigin [8]. The TFs exert structure-specific biological activities. For instance, TF3 was found to block human immunodeficiency virus-1 (HIV-1) envelope glycoprotein-mediated membrane fusion by binding with highly conserved hydrophobic pockets of the proteins to exert anti-HIV effect [9]. In an in vitro deoxyribonucleic acid (DNA) damage protective assay, TF3 appeared as a potent antioxidant compound than TF1. Furthermore, it was found that TF3 scavenges hydrogen peroxide (H_2_O_2_) and hydroxyl radical (ˉOH), while TF1 neutralizes only superoxide radicals [10]. Moreover, the monogallate ester at 3′-position played an important role in posing antioxidant effect of TFs. Compared to TF2A, TF2B potentially inhibits the superoxide radical, H_2_O_2_, and hydroxyl radical. Also, the galloyl group present in TFs is mainly responsible for the antioxidant and anticancer activity [11].

Cellular oxidative stress is generated by excessive production of reactive oxygen species (ROS), which alters the cytosolic composition by damaging biomolecules, impairing normal cellular functions leading to neurodegeneration, cancer immunosuppression, and aging [12, 13]. TFs act as a protective agent for the skin, kidney, liver, heart, and brain cells. The vast therapeutic effects of TFs include anti-inflammation, antibacterial, and anticancer, neuroprotective, antioxidant, cardioprotective, and nephroprotective [14]. TFs exert health beneficial may get effected by regulating various cellular signaling pathways particularly the activation of nuclear factor erythroid-2 related factor-2 (Nrf2)/Keap1 (Kelch-like ECH associated protein-1) signaling cascade while blocking the mitogen-activated protein kinase (MAPK) signaling to mitigate cellular inflammatory responses [15].

Considering the diverse biological potential, the present review summarizes the recent reports on the chemistry of TFs along with various associated isomers. Moreover, the pharmacological properties and clinical studies for TFs in lifestyle oriented diseases and human health are comprehensively discussed to elucidate possible mechanism of action. In addition, the effect of new formulations, including nanoformulation and encapsulation of TFs, will also be discussed to provide its modulated effect on its efficacy and bioavailability. Finally, the challenges and research gaps are discussed with future research directions.

## 2. Health Effects of TFs

TFs have been tested for its beneficial health effects and various pharmacological activities such as anticancer, skin protection, hepatoprotective, neuroprotective, anti-inflammatory, regulation of gut microbiota, antioxidant, cardioprotectant, antimicrobial, and nephroprotective effects that have been examined in both in vitro and in vivo models. These health effects are further discussed in the coming sections.

### 2.1. Anticancer Effects of TFs

TFs have extensively been studied for their anticancer affects both in vitro and in vivo cancer models. Ovarian cancer caused the highest mortalities in the cancerous gynecologic issues, and TF3 has effective role to diminish this. TF3 stimulates programmed cell death via an apoptotic pathway in the ovarian carcinoma-derived OVCAR-3 cell line [16]. TF3 increases the rate of apoptosis in rate-3 cells following a dose-dependent manner by significantly enhancing the expression of cleaved poly (ADP-ribose) polymerase 1 (PARP-1) and triggered various caspases, viz., casp-3, casp-7, casp-8, and casp-9 [16]. The casp-8 triggers downstream effector caspases responsible for the cleavage of their respective proteins, such as PARP-1. The initiation of the PARP-1 cleavage is mainly done by the caspases that initiates apoptosis by the intervention of TF3 [16, 17]. In an in vitro study, various concentrations of TF3 showed a strong but targeted effect on the growth and proliferation of human oral squamous carcinoma (HSC-2 cell line); however, no effect was seen on the normal GN46 fibroblast cells [18]. Moreover, HSC-2 cells were forced to apoptose by TF3-mediated cleavage of the PARP-1, leading to the increased expression of casp-3 levels. While, in GN46 fibroblast cells, no any alteration in the protein expression of casp-3 was seen [18]. Thus, TF3 depicted little or no harm to normal ovarian cells but combined with cisplatin, and it possesses a multifold strong antiproliferation effect against A2780/CP70 and OVCAR3 ovarian cancer cells [19]. The underlying mechanism for this combined anticancer effect of TF3 + cisplatin is the increased accumulation of platinum, and its adduct complex with DNA (Pt-DNA), which may increase DNA damage, reduced the glutathione expression with the increased expression of copper transporter 1 (CTR1) protein in the cancer cell lines [19]. Herein, TF3 may facilitate the initiation of cisplatin-induced inhibitory effects in cancer cells. The ovarian cancer stem cells (CSCs) facilitate cancer recurrence and drug resistance to lessen the long-term survival ratio in patients suffering from advanced ovarian cancer [12]. TF3 inhibited the active growth of A2780/CP70 and OVCAR3 tumorsphere cells by decreasing cell viability and colony formation capability while upregulated the protein expression of casp-3 and casp-7 in cancer cells following the Wnt/*β*-catenin signaling cascade [12].

In an in vitro study using prostate cancer cells (LNCaP), TF3 along with penta-O-galloyl-*β*-D-glucose (PGG) inhibits androgen production, which is crucial for regulating growth, differentiation, and life of the epithelial cells. Moreover, TF3, combined with PGG, inhibits rat liver microsomal 5*α*-reductase activity, reducing androgen-responsive LNCaP prostate cancer cell growth, AR production, downregulating the release of androgen-induced prostate-specific antigens, and fatty acid synthase enzyme [13].

Specific death receptors (DRs) are linked with the initiation of extrinsic apoptosis. Especially, DR-5 and Fas are the prominent representatives of DR family proteins and are considered biomarkers for most anticancer drugs. The upregulation of expression levels of DRs may dictate cancer cells for apoptosis. To counterpart the apoptotic pathways, TF3 has been reported to significantly increase DR-5 and Fas expressions in cancer cells [16]. Moreover, tumor-suppressing protein p53 shows fundamental involvement in multiple paths during anticancer activity by encouraging the intrinsic apoptotic pathway by modification of B-cell lymphoma protein 2 (Bcl-2). TF3 initiates apoptosis by upregulating p53 and proapoptotic (Bad, Bax, Puma) Bcl-2 proteins in the p53-wild-type ovarian cancer cells [20]. One other idea to combat cancer cells proliferation is to induce p53-independent apoptosis. TF3 has no direct effect on the upregulation of p53 that indicates its involvement in triggering apoptosis independent of p53 protein in ovarian carcinoma cells [16]. These facts indicate that TF3 could potentially be used in anticancer therapies to divert p53-mutant cancer cells into the apoptosis pathway.

Checkpoint kinase 2 (Chk2) enzyme acts as a key signaling molecule that transduces cellular responses to suppress tumorigenesis [21]. Upon stimulation, it indeed leads to apoptosis either without the involvement of p53 or involves p53 at multiple points [22, 23]. Any mutation or either deletion of Chk2 is linked with the oncogenesis of multiple cancers [23]. Here, the involvement of TF3 is evident with the clue that it activates the Chk2 enzyme through its upregulated phosphorylation [16]. The Chk2 arrest reduces the TF3 induced apoptosis while increasing phosphorylated Chk2 (p-Chk2), Bax, cleaved PARP-1, and activated casp-3, casp-7, and casp-9. TF3 induced reduction in the expression of B-cell lymphoma-extra-large protein (Bcl-xL). In addition, TF3- has little effect on the activation of casp-8; however, it activates Chk2, which later activates casp-9 to induce an intrinsic apoptotic cascade [24]. The mechanistic view of TFs against cancer cells has been explained in Figure 2.

### 2.2. Skin Protective Effects of TFs

Subcutaneous adipose tissue shows a vital role in skin regeneration [25]. Subcutaneous adipocytes communicate with fibroblasts and correlate with elastic fibers of the dermal skin layer and affect the structural properties of the skin layers [26, 27]. However, adipocytes become narrow with agingand decrease thermogenic power, structural stability, and dermal elasticity, contributing to skin wrinkling [28, 29]. For instance, ultraviolet radiations (UVR) caused photoaging, which can change lipid metabolism by decreasing free fatty acid and triglyceride (TG) in the adipocytes [30]. Thus, the reduced function of adipocytes affects lipid absorption in the skin and cellular consumption of the circulating free fatty acids, which induce adverse health issues like dyslipidemia [31], metabolic disorders [32], and insulin resistance [33]. TFs are recognized to influence lipid metabolism [34–36]. TFs in black tea polyphenols have an antiobesity effects in vivo using mouse models [36]. The usage of black tea reduces fat storage in the liver, reduces lipid and glucose levels, raises fecal excretion of the TGs, and diminishes adipose tissue [37]. TFs block UVR-induced photocarcinogenesis by suppressing the activity of UVR-mediated activator protein-1 (AP-1) and blockage of extracellular signals, which regulates protein kinase and c-Jun NH2-terminal kinase [38]. TF3 acts as antimelanogenic factors, which downregulate the expression levels of tyrosinase and mRNA levels [39]. TF3 primarily blocks the MAPK pathway, thereby inhibiting AP-1 formation, collagen degradation, and skin cancer (Figure 3). Black tea containing TFs may be utilized as a skin-whitening agent in the cosmetics due to its antimelanogenic effect [40]. TFs have a role in antiobesity and hypopigmentation actions and active role in lipid metabolism; however, their influence on subcutaneous tissue, especially adipocytes, is not still known [41].

### 2.3. Hepatoprotective Effects of TFs

In nonalcoholic fatty liver disease (NAFLD) (Figure 4), the liver collects massive amounts (5-10%) of fats in the absence of alcoholic usage that often leads to nonalcoholic steatohepatitis, hepatocellular carcinoma (HCC), cirrhosis, and later, in severe cases, liver transplantations are the only option [42]. Type-II diabetes, obesity, metabolic syndrome, and hyperlipidemia are the significant risk factors linked with NAFLD [43]. Usually, a healthy and nutritious diet, routine exercise, and weight loss practices are considered as better therapies for NAFLD. There is always a great desire for the quest for effective but safe pharmacotherapy to cure NAFLD.

Different drugs such as statins [44], metformin [45], polyunsaturated fatty acids [46], and pioglitazone [47] are much beneficial to cure NAFLD, but specific health issues have been reported, hence leaving a way for using natural products to cure NAFLD [48]. Several plants reported for having medicinal importance such as green tea, dark tea (Pu-erh) [49], Fuzhuan tea [50], aged Oolong tea [51], and black tea [52] have been reported to possess plenty of biologically active ingredients such as TFs, which serve as primary dietary anti-NAFLD agents [34, 53]. These anti-NAFLD molecules primarily obstruct the fatty acid synthesis pathway in the liver cells; rather, it promotes oxidation of the fatty acids (Figure 4). Moreover, reduction in the high-fat diet, which significantly causes liver inflammations and steatohepatitis, reduced adipocyte stress and increases the glucose tolerance and insulin sensitivity by focusing on various molecules in the cell, including activator of transcription 3 (STAT3), adenosine monophosphate-activated protein kinase (AMPK), acetyl-coA carboxylase (ACC), interleukin-6 (IL-6), tumor necrosis factor-*α* (TNF-*α*), phosphoglycerate mutase 1 (PGAM1), cyclooxygenase-2 (COX-2), acetyl-CoA carboxylase-*β* (ACAC-*β*), and enoyl-CoA hydratase 1 (ECHS1). TF3 is a highly potent and agile molecule in terms of reducing lipid levels in the liver cells. Numerous monomers of black tea TFs, especially TF3, reduce the lipid deposition in hepatic cells by activating the AMPK signaling pathway to prevent NAFLD by preventing prekallikrein (PK) biosynthesis and release. PK is a trypsin-related serine protease produced during proteolytic degradation of prekallikrein by the factor-XII, prolyl carboxypeptidase (PRCP), or certain intrinsic or extrinsic stimuli [54]. The pharmacological examinations highlighted that the downregulation of PK is linked with anti-inflammatory responses, controlling hypertension, recovery in cardiovascular issues, hemostasis, and improvement in metabolic activities [55]. Moreover, the suppression of PK helps reduce the lipid contents that could be of great interest in therapeutic applications for NAFLD.

In acute liver disease, the downregulation of PK prevents anti-Fas- (fatty acid synthase antibody-) mediated hepatic apoptosis and fatality [56]. TF3 is a potent inhibitor of PK and occupies its active site to make a strong check on its activities. Additionally, the suppression of PK is introduced while activating AMPK signaling cascades. These scenarios led us to assume that a TF3-PK/AMPK signaling cascade is crucial in diminishing NAFLD [57]. Also, AMPK/Akt/GSK-3*β* signaling pathway was regulated in diabetic rats and HepG2 cells when treated with *Sonchus oleraceus* Linn extracts [58]. TFs chiefly reduce the expression levels of fatty acid synthase enzyme involved in lipogenesis and showed hypolipidemic effects [59]. Also, TF3 efficiently combats OA-induced lipid accumulation in HepG2 cells. Yang and colleagues [60] demonstrated that individuals who take 3-4 cups of tea daily (200-250 g/month) could alleviate metabolic syndromes such as NAFLD to great extent.

The polyphenols present in black tea can potentially reduce the fat deposits, overall body weight, lipid biosynthesis, and obesity, which are major causes of NAFLD [61, 62]. TFs are the primary source of dietary anti-NAFLD molecules that suppress high fat-diet induced hepatic steatosis and liver inflammations. Furthermore, TFs inhibit the biosynthesis of fatty acids, upregulate their oxidation, and diminish liver and adipose tissue stress by improving glucose tolerance and insulin sensitivity through AMPK/ACC, IL-6/STAT3 signaling pathway, and TNF-*α*, COX-2, PGAM1, ACAC-*β*, and ECHS1 expression in in vivo and in vitro studies [34, 53]. In certain clinical studies, the TF enriched green tea extracts were given to 240 hypercholesterolemia patients for its lipid-lowering activity. The extracts significantly lower the total cholesterol, LDL-cholesterol, HDL-cholesterol, and triglyceride levels, with no any side effects [63]. Therefore, it can be suggested that drinking TF-based green tea could help lowering hypercholesterolemia and its associated diseases.

### 2.4. Neuroprotective Effects of TFs

The brain is the highest oxygen-consuming organ of the human body and can be impaired by ROS-mediated cellular oxidative burst and redox-activated metal ions [64]. TFs are the essential bioactive phytochemicals and native antioxidants in black tea that scavenges these free radicals. TFs have important antioxidant characteristics due to their free radical scavenging and the metal chelation property [65, 66] and hence could provide neuroprotection. Furthermore, TFs have matched in antioxidant potency to the EGCG by preventing A*β* and *α*-synuclein toxicity [67]. TFs also prevent PC12 cells from H_2_O_2_-mediated oxidative stress [68].

Additionally, TFs also inhibited 6-hydroxydopamine- (6-OHDA-) induced SH-SY5Y cell apoptosis by increasing glutathione and tyrosine hydroxylase levels, along with reduction in ROS production, and regulating the nitric oxide (NO) signaling pathway [69]. TFs also have neuroprotective effects against 1-methyl-4-phenyl-1,2,3,6-tetrahydropyridine (MPTP) toxicity that induces Parkinson's disease (PD) due to their antioxidant and antiapoptosis activities [70]. These results clearly showed that TFs could effectively prevent neurodegenerative disorders; however, indepth studies are needed comprising in vivo and clinical trials.

### 2.5. Anti-Inflammatory Effects of TFs

TFs play a vital role in eliminating inflammations (Figure 4). Cytokines such as the IL-6 expression increased during severe tissue trauma and apoptosis. TF derivatives being applied as anti-inflammatory agents and profound reduction in the IL-6 expression level were seen during viral infections [71]. Gosslau and collaborators [72] indicated that TF and TF3 specifically reduced the 12-*O*-tetradecanoylphorbol-13-acetate, which decreased the expressions of the COX-2, TNF-*α*, inducible nitric oxide synthase (iNOS), ICAM-1, and nuclear factor *κ*B (NF-*κ*B) [73]. TF3 is well known to block the phosphorylation of inhibitor of kappa B (IkB) in the cytosolic proteins and reduces the lipopolysaccharide-induced nuclear accumulation of NF*κ*B, p65, and p50 subunits [73]. Furthermore, the gallic acid moiety of TF3 is crucial for its decisive anti-inflammatory actions [73].

TFs significantly prevent the neuronal damage from cerebral ischemic repurfusion by reducing leukocyte influx and expression of ICAM-1, inhibiting the upregulation of iNOS and COX-2 in the ischemic brain by reducing the STAT-1 phosphorylation [74], Suppressing the activated epidermal growth factor receptors and reduction in mucin 5AC (MUC5AC) levels, TFs alleviate airway mucous hypersecretion which is vital in the treatment of incurable airway inflammations [75].

### 2.6. Regulation of Gut Microbial Populations by TFs

Catechins and TFs of the phenolic group possess numerous health advantages. TFs, which are derived from dimeric derivatives of catechins, have negligible bioavailability in the small intestine. TFs and their phase II metabolic substances are not identified in excreted urine 0-30 hours after consumption [76]. Hence, a significant proportion of depleted part of the catechins and TFs will penetrate the large intestine where undergoes bioconversion by residential microorganisms [77]. The gut microbiota degrades TF3 to TF1, TF2A, and TF2B [78, 79]. Later, following the degalloylation, TFs are converted to certain minor phenolic compounds like 5-(3′,4′-dihydroxy phenyl)-*γ*-valerolactone and 3-(3′,4′dihydroxyphenyl) propionic acid [76]. As like, catechins were also converted to metabolites by microbial metabolism [80]. Catechins and TFs can produce similar metabolites from microbial metabolism. This concludes that the consumption of pure catechins or TFs and green or black tea could modify the structure and metabolic actions of the gut microbiota toward a good healthy profile [81, 82]. Green or black tea intake exerted modulatory effects on gut microbiota, including growth-promoting effects on Lachnospiraceae and Akkermansia and the inhibitory effects on *Clostridium leptum* [83]. TFs and the green tea catechins have the same building blocks as flavan-3-ol. Hence, it is assumed that they form similar metabolites during fermentation of these compounds, i.e., hydroxylated phenyl carboxylic acids, a mimicking way to give modulatory effects by gut microbiota [84].

### 2.7. Antioxidant Effects of TFs

TF3 is a major and abundant ingredient in black tea, which is produced during fermentation by the reaction of epigallocatechin gallate (EGCG) and epicatechin gallate (ECG) [85]. Hence, it has been discovered that TF3 has numerous pharmacological activities, viz., anti-inflammatory and free radicals or ROS scavenging capability [65, 86] (Figure 5). A recent report pointed out that large consumption of black tea reduces the risk of aging in females [87]. Furthermore, earlier studies indicated that TF3 blocked the matrix metalloproteinase 9 (MMP-9) expression and cured calvarial osteolysis [85, 88]; hence, it prevents osteoporosis. A recent in vitro study explained that TF3 has cell-specific properties, i.e., in cancer cells and TF3 generate efflux of ROS, while on the contyrary in normal GN46 fibroblast cells, TF3 (250 *μ*M) significantly increased the levels of intracellular glutathione to provide antioxidant effects [18]. Generally, polyphenolics are widely known to exert antioxidant activity [89].

ROS play an essential role in osteoclast development and bone resorption process [90, 91]. TF3 prevents osteoclastogenesis by stimulating the Nrf2/Keap1 signaling pathway and suppressed the MAPK pathways. Furthermore, receptor activator of nuclear factor-kappa-*Β* ligand (RANKL) raises intracellular ROS level in osteoclasts which involves tumor necrosis factor receptor-associated factor 6 (TRAF6), tumor necrosis factor receptor (TNFR), Rac1, and NADPH oxidase 1 (Nox1) [90]. Meanwhile, ROS can act as a signaling molecule during RANKL in osteoclast formation [92]. Moreover, a minimum level of oxidative stress is required to increase the MAPK (ERK, JNK, p38) signaling cascades [93]. Therefore, ROS levels decreased during the development of osteoclasts by reduced antioxidant enzymes and glutathione levels, but Nrf2/Keap1 complex rescue here to diminish the oxidative stress [93]. Nrf2, a transcription factor, regulates the cytoprotective enzymes in most cells, including osteocytes, osteoclasts, and osteoblasts. Under basal conditions, Keap1 keeps Nrf2 inactive in the cytoplasm but detached from Keap1 to increase cellular oxidative stress and help translocate to the nucleus [93, 94]. Inside the nucleus, Nrf2 attaches with the antioxidant response element (ARE). Nrf2 uplifts the expression of antioxidant proteins such as heme oxygenase-1 (HO-1), catalase (CAT), glutathione peroxidase 1 (GPx1), superoxide dismutase (SOD), and phase II-detoxifying enzymes [95–97]. It indicated that antioxidant TFs decrease osteoclastogenesis and bone resorption by enhancing the expression of cytoprotective enzymes [98, 99].

### 2.8. Cardioprotective Effects of TFs

Extensive epidemiological studies reported negative correlation between tea consumption and cardiovascular diseases (CVD) [100]. Also, tea consumption is inversely associated with body mass index [101]. Tea polyphenols especially TF3 possess potent antioxidant, antiproliferative, anti-inflammatory, and antithrombotic actions [102]. Hence, dietary intake of TFs is highly recommended for persons with high cholesterol levels, obesity, heart disease, and hyperlipidemia. TF intake is inversely related to mortality from coronary heart disease.

Oxidative stress is one of the leading causes of various cardiovascular diseases, including ischemia/reperfusion (I/R) injury and atherosclerosis. Upregulation of endogenous antioxidants results in sustained cardioprotection. The reactive oxygen species (ROS), released due to oxidative stress, are partially reduced metabolites such as superoxide anions, hydroxyl radicals, hydrogen peroxide, ROS damage DNA, proteins, and lipids. Knowing these facts, proper medication using chelators [103], antioxidative [104], and antioxidants [105] improves cardiac function. They also inhibit infarction size in models of I/R injury of the heart and elevate the myocyte survival.

The extraordinary antiatherosclerotic effect of TFs has primarily been attributed to the ROS scavenging properties of TFs [106]. In addition, theaflavins possess excellent electron-donating abilities due to the hydroxyl groups in their structure [107]. TFs are thus considered efficient scavengers of free radicals such as singlet oxygen, peroxynitrite superoxide anions, and NO [108].

Dreger and coworkers [109] investigated the action of EGCG and TF3 on neonatal rat cardiomyocytes. Pretreatment with EGCG or TF3 1 h before the introduction of oxidative stress by H2O2 effectively protected cardiac myocytes as determined by measuring lactate dehydrogenase release after 24 h. H2O2-induced cellular damage was also diminished entirely. Longer preincubation times resulted in rapid loss of protection. This can be attributed to the half-life of these polyphenols in cell culture. Hence, it is concluded that both TF3 and EGCG possess potent ability to protect cardiomyocytes against oxidative stress independently of upregulation of antioxidant enzymes or activation of prosurvival kinases [110].

Endothelial cells of the arterial wall are mainly involved in inducing low-density lipoprotein (LDL) oxidation. Yoshida et al. [107] demonstrated the effect of pretreatment with tea polyphenols on the ability of cell-mediated LDL oxidation. Among all the TFs, TF3 showed the maximum inhibitory effect on the ability of cells to oxidize LDL. Parthasarathy et al. [111] also reported that TF3 attenuated the cell-mediated LDL oxidation. Pretreatment with TF3 significantly inhibited superoxide production of macrophages and chelated iron ions. Kobayashi et al. [112] demonstrated the effects of polyphenols on postprandial hypertriacylglycerolemia (HTAG) using rats. Postprandial HTAG was reported to be suppressed in a dose-dependent manner by inhibiting the pancreatic lipase enzyme. The activity of pancreatic lipase was attenuated by reducing triacylglycerol absorption. Among all TFs, TF3 showed the maximum inhibitory action against postprandial HTAG.

### 2.9. Antimicrobial Effects of TFs

TF3 has remarkable antimicrobicidal potential against *Mycoplasma salivarium*, *M. pneumonia*, and *M. orale*. Chosa et al. [113] reported the microbiocidal and antimicrobial activities of tea extracts containing TF3 and EGCG against *Mycoplasma*. *Campylobacter jejuni* (*C*. *jejuni*) is a foodborne pathogen that causes diarrhea and gastroenteritis in mammals. TFs inhibited the growth of clinical isolates of *C. coli* and *C. jejuni*. *Bacillus cereus* that is also a foodborne pathogen that leads to diarrhea and vomiting in humans [114]. The tea fractions having micro or even nanomolar concentrations of TF3 effectively inactivate *B. cereus*. The inactivation or inhibition of bacterial strains can be attributed to the ability of TF3 to bind the bacterial surface, thereby limiting the availability of receptors on the outer membrane for its attachment to the new host cells [115]. TF3 also destroys cell permeability by attacking the cell wall and cell membrane. Also, TF3 interferes and disrupts various cell functions like electron transport system, enzyme activity, nutrient uptake, proteins, and nucleic acid synthesis. All these factors lead to a retarded growth or death of bacterial cells [116] (Table 1).

Viral contamination of food is a leading cause of various infectious diseases. The mechanical approaches followed by the tea polyphenols or TFs as an antimicrobial activity are their ability to act as antioxidants, disrupt cell membranes, prevent viral binding and penetration into cells, inhibit enzymes, and trigger host cell self-defense mechanisms (Table 1). Researchers investigated that severe acute respiratory syndrome (SARS) is associated with 3CLpro, inhibited by TF3 [127]. TF3 directly influences viral particle infectivity, consistent with the inhibitory effects against the influenza virus [71]. TF3 plays a significant role in preventing HIV by attenuating the entry step [9, 128]. Hepatitis C is caused by the hepatitis C virus (HCV) [129], which may lead to liver fibrosis and cirrhosis, resulting in hepatocellular carcinoma [130]. TFs inhibit all HCV genotypes and suppress the activated viral particle. Chowdhury and colleagues [131] also reported the inhibitory action of TFs against HCV. HCV transmission between hepatocytes occurs through direct cell-to-cell transfer to infect other hepatocytes. This entry is significant for infection. Thus, this entry step is a major target for HCV inhibitors. Nowadays, entry inhibitors are given along with DAAs against HCV [132]. Zeisel and coworkers reported a synergistic effect of TFs and sofosbuvir or daclatasvir against HCV inactivation. Researchers have reported that TFs also inactivate other viruses such as HSV-1, HIV-1, and influenza virus [9, 133]. Theaflavins also possess extraordinary fungicidal activities against various fungal strains. [113]. Archana and Abraham [134] demonstrated antifungal activity of several tea extracts (green tea, fresh leaves, and black tea) against fungi such as *Aspergillus fumigates*, *Fusarium* sp., *Candida albicans*, and *Aspergillus niger.*

Certain preliminary studies for severe acute respiratory syndrome coronavirus 2 (SARS-CoV-2) 3CL-protease, the ECGC and TF were tested and found to inhibit the protease activity in a dose-dependent manner. The 3CL-protease activity is important for making functional virus proteins, which played a vital role in infection and spread. The most active dose of EGCG and TF is 7.58 *μ*g/mL and 8.44 *μ*g//mL, respectively, and was much lower than the tested toxicity dose (40 *μ*g//mL), suggested its safety over its use [135]. Also, it has been reported that both EGCG and TFs exhibited significant interactions with the target receptors of SARS-CoV-2 and thus could be a potential candidate in the treatment and prophylaxis of the COVID-19 [136].

### 2.10. TF Protective Effects on the Kidney

Acute kidney injury (AKI) is a severe health condition that results in multiple clinical issues, especially partial nephrectomy, transplantation of kidneys, severe infection, and thromboembolism of the renal artery [137]. Renal I/R is the main source of AKI [138]. Renal I/R causes a reduced supply of arterial blood in the kidneys and restores blood supply for reoxygenation. Studies have shown that the increased severity of renal I/R is associated with the generation of heavy ROS efflux, and hence programmed cell death is the fate [139, 140]. Mitochondria serve as a home for intracellular ROS, as they are byproducts of mitochondrial respiration. Renal I/R induces mitochondrial dysfunction, which triggers the production of ROS [141, 142]. Black tea polyphenols have been used widely to cure or prevent renal illnesses. Theaflavins, especially TF3, pose an inhibitory effect on serious illnesses. It reduces ROS-mediated oxidative stress by the involvement of the oxidative stress-responsive Nrf2 pathway (Figure 5). Thus, it has proven to greatly minimize the damage in brain I/R [143] and uplift radiation-mediated hematopoietic stem cells damage. Li et al. [144] developed a kidney model for I/R injury in vivo. They reported that TF3 significantly reduced the upregulation of kidney injury molecule-1 (KIM-1) in the renal tissues along with improving renal impairment lined to I/R.

Nrf2 ensures cellular redox homeostasis by regulating the expression levels of multiple oxidative stress-responsive genes. In addition, Nrf2 helps metabolize or neutralize ROS efflux and protects against cellular membranes leakage and damage of tissues in response to inflammation and oxidative stress [145]. Typically, under basal conditions, Keap1 engages Nrf2 to stay inside cytoplasm by covalent attachment, and upon the receipt of signals by redox imbalance, the former undergoes ubiquitination [146]. On the other hand, the oxidative stress or the electrophilic species can destroy the major cysteine residues in the negative regulator Keap1 to inactivate the Keap1-cullin-3 ubiquitination system. Here at this stage in the cytoplasm, Nrf2 assembles before translocating into the nucleus, where it induces transcription to a bunch of genes, particularly HO-1 and NAD(P)H dehydrogenase [quinone] encoded by quinine oxidoreductase 1 (NQO1) [145] (Figure 5). Hence, upregulation of Nrf2 to lessen oxidative stress is considered a mechanistic approach towards treating renal I/R injury [147].

Chronic renal failure (CRF) is a complete failure of the normal physiology of nephrons leading to disruption of tubules, vessels of the circulatory system, glomeruli, and renal interstitium. TFs showed a protective effect against renal failures. This preventive role can be attributed to their ability to lessen uremic toxins, production of NO, and an upregulation of the antioxidant environment in the cell. Furthermore, TFs boost the blood urea filtration process by enhancing the performance of the liver [148]. In a recent in vivo study using arginine-induced liver damage rat models, TF3 was effective against renal dysfunction [149]. This review explores the health effects of theaflavins as a pharmacological agent used for curing various illnesses (Table 2).

## 3. Effect of Formulations on TF Efficacy

The bioactivity of any drug molecule or active compound depends on its pharmacokinetics and pharmacodynamics. These properties were affected by the physicochemical characteristics of the drug molecule, and thus any modification in these characteristics could affect the bioavailability and efficacy. TFs have low bioavailability due to their high molecular weight and large polar surface area and thus require modifications before delivery [152]. Therefore, advances in formulations such as encapsulation and nanoformulations are of great importance as they increased the efficacy of the drug molecule and lower the dosage, toxicity, and other side effects.

In a nanoformulation, gold nanoparticles of TF were made and tested for their anticancer activity against human ovarian cancer cells [146]. It was interesting to see a significant improvement in the anticancer efficacy of TF gold nanoparticles compared to the bare TF. Also, the dose was significantly reduced using the nanoformulated TF. The enhanced effect was possibly due to the oxidation of TF to its quinone derivative onto the surface of gold nanoparticles, which further exerted caspase activity leading to cell death [153]. TF3 is a promising bioactive compound exerting various biological activities; however, the true value could not be harnessed due to its susceptibility to the digestion tract. To overcome this, nanoliposome encapsulated TF3 was developed and showed great in vitro digestion stability [154]. Similar to this study, another study was conducted using chitosan and casein phosphopeptides nanocomplex to encapsulate TF3 and found that the complex improved the intestinal stability and permeability of the drug [155]. In another study, natural polyphenols, such as epigallocatechin gallate (EGCG), tannic acid, curcumin, and theaflavin with previously demonstrated anticancer potential, were encapsulated into gelatin-based 200 nm nanoparticles consisting of a soft gel-like interior with or without a surrounding LbL shell of polyelectrolytes (polystyrene sulfonate/polyallylamine hydrochloride, polyglutamic acid/poly-l-lysine, dextran sulfate/protamine sulfate, carboxymethyl cellulose/gelatin, type A) assembled using the layer-by-layer technique. These polyphenolic nanocapsules found to retain its biological activity and blocked hepatocyte growth factor- (HGF-) induced intracellular signaling in the breast cancer cell line MBA-MD-231 [156]. In an interesting study, chitosan encapsulated theaflavin-enriched black tea extract (BTE) nanoparticles (ranged from 255 nm to 560 nm) were synthesized via electrospraying, and the encapsulation efficiency was recorded above 95% [157].

Overall, very few studies are conducted on TF-specific encapsulation and nanoformulations, while most studies are on the whole tea extract or polyphenolic extract [158–160]. Therefore, it would be suggested that more research on formulations needs to be conducted to improve TFs bioavailability, efficacy, and gastrointestinal stability.

## 4. Conclusion

The current review summarized the health effects of TFs and their underlying mechanisms. TF1, TF2A, TF2B, and TF3 are the major TF derivatives reported for a wide range of biological activities. Among these, TF3 is largely studied for its biological effects such as antioxidant, anti-inflammatory, anticancer, and antimicrobial activities. Among all these activities, the anticancer effect of TFs was largely studied both in in vitro and in vivo models. Also, synergistic activity of TFs was reported when used in combination with other drugs. The anticancer activity of TFs was mainly exerted by triggering the caspases, skin protection effect by blocking the MAPK pathway, hepatoprotection by activating AMPK pathway, neuroprotective by regulating NO signaling, reduce inflammations by upregulation of inflammation-linked prooxidative enzymes, cardioprotective by ROS scavenging and by preventing cell-mediated LDL oxidation, and exerted kidney protective effect by downregulating the KIM-1. Although a large number of in vitro and in vivo studies on the TFs effect are available, however, very few studies are available on its clinical efficacy and thus limit its overall use. Also, the new formulations (nanoformulation/encapsulation) have been developed to modify the TF bioavailability and efficacy that has shown promising results. The current research on TF biological activities clearly showed its extended use in clinical trials and thus recommended for future studies. Also, more data needs to be conducted to develop new formulations to provide a better drug candidate (higher bioavailability and efficacy).

## Figures and Tables

**Figure 1:** Structural diversity in theaflavins.

**Figure 2:** The mechanism of anticancer activity of theaflavins (TFs). TFs follow multiple pathways to induce apoptosis in cancer cells.

**Figure 3:** The cytoprotective mechanism of TFs in skin cells against solar UVR by inhibiting ROS-mediated MAPK signaling cascades.

**Figure 4:** The TFs downregulate nonalcoholic fatty liver disease (NAFLD) and its associated risk factors and regulates the biosynthesis of unnecessary fatty acids in liver cells. Moreover, glucose tolerance and insulin sensitivity have also been increased. NASH: nonalcoholic steatohepatitis; HCC: hepatocellular carcinoma, cirrhosis; AMPK: adenosine monophosphate-activated protein kinase; PK: plasma kallikrein.

**Figure 5:** The regulation of antioxidant responsive Nrf2/HO-1 pathway to combat ROS mediated renal cell injury and provides cytoprotection by reducing the production of inflammatory mediators.

**Table 1:** Inhibitory activity of tea TFs against pathogenic and spoilage bacteria, viruses, and fungi.

Organism	Class	Adverse effects	Inhibitors	References
Human immunodeficiency	Virus	AIDS	Theaflavins	[9, 117–119]
Cholera	Toxin	Cholera	Theaflavins	[120–122]
Antihemolysin *α*-toxin	Bacteria	Infections	Theaflavins	[120, 122]
Phytopathogens	Bacteria	Plant disease	Theaflavins	[123]
*Bo. pertussis*	Bacteria	Whooping cough	TF3	[124]
*Ba. cereus*	Bacteria	Food poisoning; emesis	Theaflavins	[125, 126]

**Table 2:** The pharmacological activities of theaflavin and its derivatives.

Theaflavins	In vitro/in vivo model	Results	Refs
TF3	Human ovarian cancer cells (A2780/CP70 and OVCAR3 cells)	Decreasing cell viability and upregulating the protein expression of caspase-3 and -7 in the cells	[12]
TF3 and (PGG)	LNCaP prostate cancer cells	Reduced androgen-responsive LNCaP prostate cancer cell growth, suppressed expression of the AR	[13]
TF3	Human ovarian cancer cells (OVCAR-3)	Activate extrinsic apoptosis in OVCAR-3 cells by inducing G0/G1 cell cycle arrest	[16]
TF-3	Human oral squamous carcinoma HSC-2 cells and normal GN46 fibroblasts	Induction of apoptotic cell death by elevated activity of caspase-3	[18]
TF3 and cisplatin	Human ovarian cancer cells (A2780/CP70 and OVCAR3 cells)	Combined treatment showed a synergistic cytotoxicity	[19]
TF3	Cisplatin-resistant ovarian cancer A2780/CP70 cells	G2 cell cycle arrest	[20]
Theaflavins (TF-1, TF-2, TF-3)	HepG2 cells, cell culture, and high-fat dietMale Wistar rats	Reduced lipid accumulation, suppressed fatty acid synthesis, and stimulated fatty acid oxidation	[34]
Theaflavins, EGCG	JB6 mouse epidermal cell line	Both inhibited UVB-induced AP-1 activation. Inhibitory effects of theaflavins were stronger than those of EGCG	[38]
TF-3	*α* Melanocyte-stimulating hormone (*α*MSH)-induced melanogenesis in mouse B16 melanoma cells	Showed inhibitory effect on melanogenesis due to suppression of tyrosinase protein and mRNA levels	[39]
Cofermented green tea with a high level of TFs	Human subcutaneous fat cells (hSCFs)	Promoted differentiation of hSCFs	[41]
Theaflavin	Mouse fatty liver model	Decreased liver steatosis, oxidative stress, inflammation, and hepatocyte apoptosis	[53]
TF3	HepG2 cells and HEK 293T cells	Reduced lipid droplet accumulation in hepatocytes, inhibited the activation of plasma kallikrein, and stimulate AMPK	[57]
TF1, TF2A, TF2B and TF3	Cell model of PC12 cells	Prevent oxidative stress by suppressing oxidant enzyme activity and downregulated the expression of caspase-3	[68]
TFs	Human neuroblastoma SH-SY5Y cells	Prevented 6-hydroxydopamine-induced loss of cell viability, condensed nuclear morphology, and apoptosis	[69]
TFs	MPTP/p induced neurodegenaration in C57BL/6 mice	Attenuates apoptosis and neurodegeneration	[70]
TFs	Influenza virus in vitro	Inhibitory effects against influenza virus	[71]
TF-2	Human colon cancer cells	Induced the upregulation of *P53* and *BAX*and suppressed the *COX-2* gene expression and also downregulated TNF-*α*, iNOS, ICAM-1, and NF*κ*B	[72]
Theaflavin	Cerebral I/R injury in rats	Inhibited leukocyte infiltration and expression of ICAM-1, COX-2, and iNOS. Suppressing upregulation of iNOS and COX-2	[74]
TF3	Male C57BL/6 mice, bone marrow-derived macrophages and RAW264.7 murine acrophages	Inhibited osteolysis and prevented bone destruction. Suppressed osteoclast formation, polarization and osteoclastic bone resorption	[85]
TF3	Acute lung injury (ALI) in a mouse model. RAW 264.7 macrophages	Suppressed the phosphorylation of c-Jun N-terminal kinase and p38 MAPK,TNF-*α*, IL-1, and IL-6	[86]
TF1, TF2A, TF2B and TF3	Herpes simplex virus type 1 infected Vero and A549 cells	TF3 showed most strong anti-HSV-1 effect in both Vero and A549 cells	[133]
Theaflavin	C57/BL6 J model of I/R injury, hypoxia/reoxygenation (H/R) model of TCMK-1 cells	Inhibited I/R- and H/R-induced renal injury and cell apoptosis	[144]
Theaflavins and thearubigins	Arginine induced renal alfunction in rats	Significant reduction in lipid profile, glucose content, renal function tests and TBARS with enhancement in insulin, HDL, and hematological parameters	[149]
Catechins, theaflavins	C3(1) SV40 T,t antigen transgenic mouse model	The size of the largest tumor per mouse was decreased. Increased levels of cleaved caspase-3 in tumor tissue and increased apoptosis.	[150]
Mixture of TF3, TF2A, TF2B thearubigin, and EGCG	Lipopolysaccharide-activated murine macrophages, RAW 264.7 cells	TF3 exerted strong inhibiting effect on NO generation than EGCG	[151]

## Data Availability

All data used to support the findings of this study are included in the paper.

## Abbreviations

TFs: Theaflavins
TF1: Theaflavin
TF2A: Theaflavin-3-gallate
TF2B: Theaflavin-3′-gallate
TF3: Theaflavin-3,3′-digallate
ROS: Reactive oxygen species
Nrf2: Nuclear factor erythroid-2 related factor-2
Keap1: Kelch-like ECH associated protein-1
MAPK: Mitogen-activated protein kinase
PARP-1: Poly (ADP-ribose) polymerase 1
CTR1: Copper transporter 1
CSCs: Cancer stem cells
PGG: Penta-O-galloyl-*β*-D-glucose
DNA: Deoxyribonucleic acid
DRs: Specific death receptors
Chk2: Checkpoint kinase 2
Bcl-xL: B-cell lymphoma-extra-large protein
TG: Triglyceride
UVR: Ultra violet radiation
NAFLD: Non-alcoholic fatty liver disease
HCC: hepatocellular carcinoma
AMPK: Adenosine monophosphate-activated protein kinase
ACC: Acetyl-coA carboxylase
IL-6: Interleukin-6
TNF-*α*: Tumor necrosis factor-*α*
PGAM1: Phosphoglycerate mutase 1
ACAC-*β*: Acetyl-CoA carboxylase-*β*
ECHS1: Enoyl-CoA hydratase 1
PRCP: Prolyl carboxypeptidase
6-OHDA: 6-Hydroxydopamine
MPTP: 1-Methyl-4-phenyl-1,2,3,6-tetrahydropyridine
PD: Parkinson's disease
COX-2: Cyclooxygenase-2
iNOS: Inducible nitric oxide synthase
ICAM-1: Intercellular Adhesion Molecule 1
NF-*κ*B: Nuclear factor *κ*appa B
IkB: Inhibitor of kappa B
STAT-1: Signal transducer and activator of transcription 1
STAT3: Signal transducer and activator of transcription 3
EGCG: Epigallocatechin gallate
ECG: Epicatechin gallate
MMP-9: Matrix metalloproteinase 9
RANKL: Receptor activator of nuclear factor-kappa-*Β* ligand
TRAF6: Tumor necrosis factor receptor-associated factor 6
TNFR: Tumor necrosis factor receptor
Nox1: NADPH oxidase 1
ARE: Antioxidant response element
HO-1: Heme oxygenase-1
CAT: Catalase
GPx1: Glutathione peroxidase 1
SOD: Superoxide dismutase
CVD: Cardiovascular diseases
LDL: Low-density lipoprotein
HTAG: Hypertriacylglycerolemia
SARS: Severe acute respiratory syndrome
HCV: Hepatitis C virus
SARS-CoV-2: Severe acute respiratory syndrome coronavirus 2
AKI: Acute kidney injury
NQO1: NAD(P)H dehydrogenase [quinone] encoded by quinine oxidoreductase 1
CRFV: Chronic renal failure
COVID-19: Coronavirus disease
HSV-1: Herpes simplex virus 1
HIV: Human immunodeficiency virus
H_2_O_2_: hydrogen peroxide.

## References

[1] Anderson R. (2014). Tea industry’s future depends on corporate collaboration. *BBC News Business*.

[2] Webster N. (1981). *Webster's Third New International Dictionary of the English Language, Unabridged, vol. 1*.

[3] Workman D. (2019). *Tea Exports by Country*.

[4] Bolton D. (2016). *Global Tea Production 2015*.

[5] Fatima M., Kesharwani R. K., Misra K., Rizvi S. I. (2013). Protective effect of theaflavin on erythrocytes subjected to In Vitro oxidative stress. *Biochemistry Research International*.

[6] Subramanian N., Venkatesh P., Ganguli S., Sinkar V. P. (1999). Role of polyphenol oxidase and peroxidase in the generation of black tea theaflavins. *Journal of Agricultural and Food Chemistry*.

[7] Tanaka T., Mine C., Inoue K., Matsuda M., Kouno I. (2002). Synthesis of theaflavin from epicatechin and epigallocatechin by plant homogenates and role of epicatechin quinone in the synthesis and degradation of theaflavin. *Journal of Agricultural and Food Chemistry*.

[8] Hodgson J. M. (2008). Tea flavonoids and cardiovascular disease. *Asia Pacific Journal of Clinical Nutrition*.

[9] Liu S., Lu H., Zhao Q. (2005). Theaflavin derivatives in black tea and catechin derivatives in green tea inhibit HIV-1 entry by targeting gp41. *Biochimica et Biophysica Acta (BBA)-General Subjects*.

[10] Wu Y.-Y., Li W., Xu Y., Jin E. H., Tu Y. Y. (2011). Evaluation of the antioxidant effects of four main theaflavin derivatives through chemiluminescence and DNA damage analyses. *Journal of Zhejiang University Science B*.

[11] Tan Q., Peng L., Huang Y. (2019). Structure–activity relationship analysis on antioxidant and anticancer actions of Theaflavins on human colon cancer cells. *Journal of Agricultural and Food Chemistry*.

[12] Pan H., Kim E., Rankin G. O., Rojanasakul Y., Tu Y., Chen Y. C. (2018). Theaflavin-3,3′-digallate inhibits ovarian cancer stem cells via suppressing Wnt/*β*-Catenin signaling pathway. *Journal of Functional Foods*.

[13] Lee H.-H., Ho C.-T., Lin J.-K. (2004). Theaflavin-3,3′-digallate and penta-O-galloyl- -D-glucose inhibit rat liver microsomal 5 -reductase activity and the expression of androgen receptor in LNCaP prostate cancer cells. *Carcinogenesis*.

[14] Rohini S., Vishnupriya P., Rakshagan V., Jain A. R. (2018). Protective effects of theaflavin. *Drug Invent Today*.

[15] Liu W., Li J. (2019). Theaflavin-3, 3′-digallate attenuates rheumatoid inflammation in mice through the nuclear factor-*κ*B and MAPK pathways. *Archivum Immunologiae et Therapiae Experimentalis*.

[16] Gao Y., Yin J., Tu Y., Chen Y. (2019). Theaflavin-3, 3′-digallate suppresses human ovarian carcinoma OVCAR-3 cells by regulating the checkpoint kinase 2 and p27 kip1 pathways. *Molecules*.

[17] Chaitanya G. V., Alexander J. S., Babu P. P. (2010). PARP-1 cleavage fragments: signatures of cell-death proteases in neurodegeneration. *Cell Communication and Signaling*.

[18] Schuck A. G., Ausubel M. B., Zuckerbraun H. L., Babich H. (2008). Theaflavin-3,3′-digallate, a component of black tea: An inducer of oxidative stress and apoptosis. *Toxicology In Vitro*.

[19] Pan H., Kim E., Rankin G., Rojanasakul Y., Tu Y., Chen Y. (2018). Theaflavin-3, 3′-Digallate enhances the inhibitory effect of cisplatin by regulating the copper transporter 1 and glutathione in human ovarian cancer cells. *International Journal of Molecular Sciences*.

[20] Tu Y., Kim E., Gao Y., Rankin G. O., Li B., Chen Y. C. (2016). Theaflavin-3, 3′-digallate induces apoptosis and G2 cell cycle arrest through the Akt/MDM2/p53 pathway in cisplatin-resistant ovarian cancer A2780/CP70 cells. *International Journal of Oncology*.

[21] Nevanlinna H., Bartek J. (2006). The _CHEK2_ gene and inherited breast cancer susceptibility. *Oncogene*.

[22] Powers J. T., Hong S., Mayhew C. N., Rogers P. M., Knudsen E. S., Johnson D. G. (2004). E2F1 uses the ATM signaling pathway to induce p53 and Chk2 phosphorylation and apoptosis11American Cancer Society (ES Knudsen) and NIH (grants CA98601, ES11047, ES07784, CA16672, and T32ESO7247). *Molecular Cancer Research*.

[23] Urist M. (2004). p73 induction after DNA damage is regulated by checkpoint kinases Chk1 and Chk2. *Genes & Development*.

[24] Gurley K. E., Moser R., Gu Y., Hasty P., Kemp C. J. (2009). DNA-PK suppresses a p53-independent apoptotic response to DNA damage. *EMBO Reports*.

[25] Kruglikov I. L., Scherer P. E. (2016). Skin aging: are adipocytes the next target?. *Aging*.

[26] Ezure T., Amano S. (2015). Increment of subcutaneous adipose tissue is associated with decrease of elastic fibres in the dermal layer. *Experimental Dermatology*.

[27] Mukhtar H., Ahmad N. (2000). Tea polyphenols: prevention of cancer and optimizing health. *The American Journal of Clinical Nutrition*.

[28] Kruglikov I. L., Scherer P. E. (2017). General theory of skin reinforcement. *PLoS One*.

[29] Pawlaczyk M., Lelonkiewicz M., Wieczorowski M. (2013). Age-dependent biomechanical properties of the skin. *Advances in Dermatology and Allergology/Postȩpy Dermatologii i Alergologii*.

[30] Kim E. J., Kim Y. K., Kim J. E. (2011). UV modulation of subcutaneous fat metabolism. *Journal of Investigative Dermatology*.

[31] Lemieux I. (2004). Energy partitioning in gluteal-femoral fat: does the metabolic fate of triglycerides affect coronary heart disease risk?. *Arteriosclerosis, Thrombosis, and Vascular Biology*.

[32] Miranda P. J., DeFronzo R. A., Califf R. M., Guyton J. R. (2005). Metabolic syndrome: definition, pathophysiology, and mechanisms. *American Heart Journal*.

[33] Petrofsky J. S., Prowse M., Lohman E. (2008). The influence of ageing and diabetes on skin and subcutaneous fat thickness in different regions of the body. *Journal of Applied Reliability*.

[34] Lin C.-L., Huang H.-C., Lin J.-K. (2007). Theaflavins attenuate hepatic lipid accumulation through activating AMPK in human HepG2 cells^s⃞^. *Journal of Lipid Research*.

[35] Pan H., Gao Y., Tu Y. (2016). Mechanisms of body weight reduction by black tea polyphenols. *Molecules*.

[36] Yamashita Y., Wang L., Wang L., Tanaka Y., Zhang T., Ashida H. (2014). Oolong, black and pu-erh tea suppresses adiposity in mice via activation of AMP-activated protein kinase. *Food & Function*.

[37] Hamdaoui M. H., Snoussi C., Dhaouadi K. (2016). Tea decoctions prevent body weight gain in rats fed high-fat diet; black tea being more efficient than green tea. *Journal of Nutrition & Intermediary Metabolism*.

[38] Nomura M., Ma W. Y., Huang C. (2000). Inhibition of ultraviolet B–induced AP-1 activation by theaflavins from black tea. *Molecular Carcinogenesis*.

[39] Yamaoka Y., Ohguchi K., Itoh T., Nozawa Y., Akao Y. (2009). Effects of theaflavins on melanin biosynthesis in mouse B16 melanoma cells. *Bioscience, Biotechnology, and Biochemistry*.

[40] Kim Y. C., Choi S. Y., Park E. Y. (2015). Anti-melanogenic effects of black, green, and white tea extracts on immortalized melanocytes. *Journal of Veterinary Science*.

[41] Park P. J., Rha C.-S., Kim S. T. (2019). Theaflavin-enriched fraction stimulates adipogenesis in human subcutaneous fat cells. *International Journal of Molecular Sciences*.

[42] Brunt E. M., Wong V. W. S., Nobili V. (2015). Nonalcoholic fatty liver disease. *Nature Reviews Disease Primers*.

[43] Stefan N., Häring H.-U., Cusi K. (2019). Non-alcoholic fatty liver disease: causes, diagnosis, cardiometabolic consequences, and treatment strategies. *The lancet Diabetes & Endocrinology*.

[44] Sattar N., Forrest E., Preiss D. (2014). Non-alcoholic fatty liver disease. *BMJ*.

[45] Sundelin E. I. O., Gormsen L. C., Heebøll S. (2019). Hepatic exposure of metformin in patients with non-alcoholic fatty liver disease. *British Journal of Clinical Pharmacology*.

[46] Jump D. B., Lytle K. A., Depner C. M., Tripathy S. (2018). Omega-3 polyunsaturated fatty acids as a treatment strategy for nonalcoholic fatty liver disease. *Pharmacology & Therapeutics*.

[47] Xu P., Zhang X. G., Li Y. M., Yu C. H., Xu L., Xu G. Y. (2006). Research on the protection effect of pioglitazone for non-alcoholic fatty liver disease (NAFLD) in rats. *Journal of Zhejiang University Science B*.

[48] Bagherniya M. (2018). Medicinal plants and bioactive natural compounds in the treatment of non- alcoholic fatty liver disease: A clinical review. *Pharmacological Research*.

[49] Cai X., Fang C., Hayashi S. (2016). Pu-erh tea extract ameliorates high-fat diet-induced nonalcoholic steatohepatitis and insulin resistance by modulating hepatic IL-6/STAT3 signaling in mice. *Journal of Gastroenterology*.

[50] Liu Z., Lin Y., Zhang S., Wang D., Liang Q., Luo G. (2015). Comparative proteomic analysis using 2DE-LC-MS/MS reveals the mechanism of Fuzhuan brick tea extract against hepatic fat accumulation in rats with nonalcoholic fatty liver disease. *Electrophoresis*.

[51] Yuan E., Duan X., Xiang L. (2018). Aged oolong tea reduces high-fat diet-induced fat accumulation and dyslipidemia by regulating the AMPK/ACC signaling pathway. *Nutrients*.

[52] Eguchi T., Kumagai C., Fujihara T., Takemasa T., Ozawa T., Numata O. (2013). Black tea high-molecular-weight polyphenol stimulates exercise training-induced improvement of endurance capacity in mouse via the link between AMPK and GLUT4. *PLoS One*.

[53] Luo X.-Y., Takahara T., Hou J. (2012). Theaflavin attenuates ischemia-reperfusion injury in a mouse fatty liver model. *Biochemical and Biophysical Research Communications*.

[54] Kolte D., Shariat-Madar Z. (2016). Plasma kallikrein inhibitors in cardiovascular disease. *Cardiology in Review*.

[55] Feener E. P., Zhou Q., Fickweiler W. (2013). Role of plasma kallikrein in diabetes and metabolism. *Thrombosis and Haemostasis*.

[56] Li M., Qin X. Y., Furutani Y. (2018). Prevention of acute liver injury by suppressing plasma kallikrein-dependent activation of latent TGF-*β*. *Biochemical and Biophysical Research Communications*.

[57] Zhang W., An R., Li Q. (2020). Theaflavin TF3 relieves hepatocyte lipid deposition through activating an AMPK signaling pathway by targeting plasma Kallikrein. *Journal of Agricultural and Food Chemistry*.

[58] Chen L., Lin X., Fan X., Qian Y., Lv Q., Teng H. (2020). *Sonchus oleraceus* Linn extract enhanced glucose homeostasis through the AMPK/Akt/ GSK-3 *β* signaling pathway in diabetic liver and HepG2 cell culture. *Food and Chemical Toxicology*.

[59] Yeh C., Chen W. J., Chiang C. T., Lin-Shiau S. Y., Lin J. K. (2003). Suppression of fatty acid synthase in MCF-7 breast cancer cells by tea and tea polyphenols: a possible mechanism for their hypolipidemic effects. *The Pharmacogenomics Journal*.

[60] Yang C. S., Zhang J. (2019). Studies on the prevention of cancer and cardiometabolic diseases by tea: issues on mechanisms, effective doses, and toxicities. *Journal of Agricultural and Food Chemistry*.

[61] Pan S., Deng X., Sun S. (2018). Black tea affects obesity by reducing nutrient intake and activating AMP-activated protein kinase in mice. *Molecular Biology Reports*.

[62] Park B., Lee S., Lee B. (2016). New ethanol extraction improves the anti-obesity effects of black tea. *Archives of Pharmacal Research*.

[63] Maron D. J., Lu G. P., Cai N. S. (2003). Cholesterol-lowering effect of a theaflavin-enriched green tea Extract. *Archives of Internal Medicine*.

[64] Valko M., Leibfritz D., Moncol J., Cronin M. T. D., Mazur M., Telser J. (2007). Free radicals and antioxidants in normal physiological functions and human disease. *The International Journal of Biochemistry & Cell Biology*.

[65] Leung L. K., Su Y., Chen R., Zhang Z., Huang Y., Chen Z. Y. (2001). Theaflavins in black tea and catechins in green tea are equally effective antioxidants. *The Journal of Nutrition*.

[66] Miller N. J., Castelluccio C., Tijburg L., Rice-Evans C. (1996). The antioxidant properties of theaflavins and their gallate esters—radical scavengers or metal chelators?. *FEBS Letters*.

[67] Grelle G., Otto A., Lorenz M., Frank R. F., Wanker E. E., Bieschke J. (2011). Black tea theaflavins inhibit formation of toxic amyloid-*β* and *α*-synuclein fibrils. *Biochemistry*.

[68] Zhang J., Cai S., Li J. (2016). Neuroprotective effects of theaflavins against oxidative stress-induced apoptosis in PC12 cells. *Neurochemical Research*.

[69] Luo Z., Zhao Y., Wang Y., Yang X., Zhao B. (2012). Protective effect of theaflavins on neuron against 6-hydroxydopamine-induced apoptosis in SH-SY5Y cells. *Journal of Clinical Biochemistry and Nutrition*.

[70] Anandhan A., Tamilselvam K., Radhiga T., Rao S., Essa M. M., Manivasagam T. (2012). Theaflavin, a black tea polyphenol, protects nigral dopaminergic neurons against chronic MPTP/probenecid induced Parkinson's disease. *Brain Research*.

[71] Zu M., Yang F., Zhou W., Liu A., du G., Zheng L. (2012). _In vitro_ anti-influenza virus and anti-inflammatory activities of theaflavin derivatives. *Antiviral Research*.

[72] Gosslau A., En Jao D. L., Huang M. T. (2011). Effects of the black tea polyphenol theaflavin-2 on apoptotic and inflammatory pathwaysin vitroandin Vivo. *Molecular Nutrition & Food Research*.

[73] Lin Y.-L., Tsai S. H., Lin-Shiau S. Y., Ho C. T., Jen-Kun Lin (1999). Theaflavin-3,3′-digallate from black tea blocks the nitric oxide synthase by down-regulating the activation of NF-*κ*B in macrophages. *European Journal of Pharmacology*.

[74] Cai F., Li C. R., Wu J. L. (2006). Theaflavin ameliorates cerebral ischemia-reperfusion injury in rats through its anti-inflammatory effect and modulation of STAT-1. *Mediators of Inflammation*.

[75] Wu H., Li Q., Zhou X., Kolosov V. P., Perelman J. M. (2012). Theaflavins extracted from black tea inhibit airway mucous hypersecretion induced by cigarette smoke in rats. *Inflammation*.

[76] Pereira-Caro G., Moreno-Rojas J. M., Brindani N. (2017). Bioavailability of black tea theaflavins: absorption, metabolism, and colonic catabolism. *Journal of Agricultural and Food Chemistry*.

[77] Cueva C., Gil-Sánchez I., Ayuda-Durán B. (2017). An integrated view of the effects of wine polyphenols and their relevant metabolites on gut and host health. *Molecules*.

[78] Chen H., Parks T. A., Chen X., Gillitt N. D., Jobin C., Sang S. (2011). Structural identification of mouse fecal metabolites of theaflavin 3,3′-digallate using liquid chromatography tandem mass spectrometry. *Journal of Chromatography A*.

[79] Chen H., Hayek S., Rivera Guzman J. (2012). The microbiota is essential for the generation of black tea theaflavins-derived metabolites. *PLoS One*.

[80] Chen H., Sang S. (2014). Biotransformation of tea polyphenols by gut microbiota. *Journal of Functional Foods*.

[81] Chen T., Liu A. B., Sun S. (2019). Green tea polyphenols modify the gut microbiome indb/dbMice as co-abundance groups correlating with the blood glucose lowering effect. *Molecular Nutrition & Food Research*.

[82] Liu Z., Bruins M. E., Ni L., Vincken J. P. (2018). Green and black tea phenolics: bioavailability, transformation by colonic microbiota, and modulation of colonic microbiota. *Journal of Agricultural and Food Chemistry*.

[83] Liu Z., Chen Z., Guo H. (2016). The modulatory effect of infusions of green tea, oolong tea, and black tea on gut microbiota in high-fat-induced obese mice. *Food & Function*.

[84] Liu Z., de Bruijn W. J., Bruins M. E., Vincken J. P. (2021). Microbial metabolism of theaflavin-3, 3′-digallate and its gut microbiota composition modulatory effects. *Journal of Agricultural and Food Chemistry*.

[85] Hu X., Ping Z., Gan M. (2017). Theaflavin-3,3′-digallate represses osteoclastogenesis and prevents wear debris-induced osteolysis via suppression of ERK pathway. *Acta Biomaterialia*.

[86] Wu Y., Jin F., Wang Y. (2017). In vitro and in vivo anti-inflammatory effects of theaflavin-3,3′-digallate on lipopolysaccharide-induced inflammation. *European Journal of Pharmacology*.

[87] Oka Y., Iwai S., Amano H. (2012). Tea polyphenols inhibit rat osteoclast formation and differentiation. *Journal of Pharmacological Sciences*.

[88] Myers G., Prince R. L., Kerr D. A. (2015). Tea and flavonoid intake predict osteoporotic fracture risk in elderly Australian women: a prospective study. *The American Journal of Clinical Nutrition*.

[89] Teng H., Fang T., Lin Q., Song H., Liu B., Chen L. (2017). Red raspberry and its anthocyanins: bioactivity beyond antioxidant capacity. *Trends in Food Science & Technology*.

[90] Lee N. K., Choi Y. G., Baik J. Y. (2005). A crucial role for reactive oxygen species in RANKL-induced osteoclast differentiation. *Blood*.

[91] Chen K., Qiu P., Yuan Y. (2019). Pseurotin a inhibits osteoclastogenesis and prevents ovariectomized-induced bone loss by suppressing reactive oxygen species. *Theranostics*.

[92] Ha H., Bok Kwak H., Woong Lee S. (2004). Reactive oxygen species mediate RANK signaling in osteoclasts. *Experimental Cell Research*.

[93] Hyeon S., Lee H., Yang Y., Jeong W. (2013). Nrf2 deficiency induces oxidative stress and promotes RANKL-induced osteoclast differentiation. *Free Radical Biology & Medicine*.

[94] Kobayashi A., Kang M. I., Okawa H. (2004). Oxidative stress sensor Keap1 functions as an adaptor for Cul3-based E3 ligase to regulate proteasomal degradation of Nrf2. *Molecular and Cellular Biology*.

[95] Park C. K., Lee Y., Kim K. H., Lee Z. H., Joo M., Kim H. H. (2014). Nrf2 is a novel regulator of bone acquisition. *Bone*.

[96] Sun Y.-X., Xu A. H., Yang Y., Li J. (2015). Role of Nrf2 in bone metabolism. *Journal of Biomedical Science*.

[97] Tu W., Wang H., Li S., Liu Q., Sha H. (2019). The anti-inflammatory and anti-oxidant mechanisms of the Keap1/Nrf2/ARE signaling pathway in chronic diseases. *Aging and Disease*.

[98] Lee S.-H., Kim J.-K., Jang H.-D. (2014). Genistein inhibits osteoclastic differentiation of RAW 264.7 cells via regulation of ROS production and scavenging. *International Journal of Molecular Sciences*.

[99] Kanzaki H., Katsumata Y., Itohiya K. (2018). Dimethyl fumarate inhibits osteoclasts via attenuation of reactive oxygen species signalling by augmented antioxidation. *Journal of Cellular and Molecular Medicine*.

[100] Geleijnse J. M., Launer L. J., van der Kuip D. A. M., Hofman A., Witteman J. C. M. (2002). Inverse association of tea and flavonoid intakes with incident myocardial infarction: the Rotterdam study. *The American Journal of Clinical Nutrition*.

[101] Vernarelli J. A., Lambert J. D. (2013). Tea consumption is inversely associated with weight status and other markers for metabolic syndrome in US adults. *European Journal of Nutrition*.

[102] Stangl V., Dreger H., Stangl K., Lorenz M. (2007). Molecular targets of tea polyphenols in the cardiovascular system. *Cardiovascular Research*.

[103] vanden Hoek T. L., Shao Z., Li C., Zak R., Schumacker P. T., Becker L. B. (1996). Reperfusion injury on cardiac myocytes after simulated ischemia. *American Journal of Physiology-Heart and Circulatory Physiology*.

[104] Chen Z., Siu B., Ho Y. S. (1998). Overexpression of MnSOD protects against myocardial ischemia/reperfusion injury in transgenic mice. *Journal of Molecular and Cellular Cardiology*.

[105] Horwitz L. D., Fennessey P. V., Shikes R. H., Kong Y. (1994). Marked reduction in myocardial infarct size due to prolonged infusion of an antioxidant during reperfusion. *Circulation*.

[106] Urquiaga I., Leighton F. (2000). Plant polyphenol antioxidants and oxidative stress. *Biological Research*.

[107] Yoshida H., Ishikawa T., Hosoai H. (1999). Inhibitory effect of tea flavonoids on the ability of cells to oxidize low density lipoprotein. *Biochemical Pharmacology*.

[108] Jovanovic S. V., Simic M. G. (2000). Antioxidants in nutrition. *Annals of the New York Academy of Sciences*.

[109] Dreger H., Lorenz M., Kehrer A., Baumann G., Stangl K., Stangl V. (2008). Characteristics of catechin-and theaflavin-mediated cardioprotection. *Experimental Biology and Medicine*.

[110] Hong J., Lu H., Meng X., Ryu J. H., Hara Y., Yang C. S. (2003). Stability, cellular uptake, biotransformation, and efflux of tea polyphenol (−)-epigallocatechin-3-gallate in HT-29 human colon adenocarcinoma cells. *Cancer Research*.

[111] Parthasarathy S. (1992). Evidence for an additional intracellular site of action of probucol in the prevention of oxidative modification of low density lipoprotein. Use of a new water-soluble probucol derivative. *The Journal of Clinical Investigation*.

[112] Kobayashi M., Ichitani M., Suzuki Y. (2009). Black-tea polyphenols suppress postprandial hypertriacylglycerolemia by suppressing lymphatic transport of dietary fat in rats. *Journal of Agricultural and Food Chemistry*.

[113] Friedman M. (2007). Overview of antibacterial, antitoxin, antiviral, and antifungal activities of tea flavonoids and teas. *Molecular Nutrition & Food Research*.

[114] Diker K., Akan M., Hascelik G., Yurdakök M. (1991). The bactericidal activity of tea against campylobacter jejuni and campylobacter coli. *Letters in Applied Microbiology*.

[115] Padmini E., Valarmathi A., Rani M. U. (2010). Comparative analysis of chemical composition and antibacterial activities of Mentha spicata and Camellia sinensis. *Asian Journal of Experimental Biological Sciences*.

[116] Zhang Y.-M., White S. W., Rock C. O. (2006). Inhibiting Bacterial Fatty Acid Synthesis. *Journal of Biological Chemistry*.

[117] Yamaguchi K., Honda M., Ikigai H., Hara Y., Shimamura T. (2002). Inhibitory effects of (−)-epigallocatechin gallate on the life cycle of human immunodeficiency virus type 1 (HIV-1). *Antiviral Research*.

[118] Hamza A., Zhan C.-G. (2006). How can (−)-epigallocatechin gallate from green tea prevent HIV-1 infection? Mechanistic insights from computational modeling and the implication for rational design of anti-HIV-1 entry inhibitors. *The Journal of Physical Chemistry B*.

[119] Kawai K., Tsuno N. H., Kitayama J. (2003). Epigallocatechin gallate, the main component of tea polyphenol, binds to CD4 and interferes with gp120 binding. *Journal of Allergy and Clinical Immunology*.

[120] Ganguly N., Kaur T. (1996). Mechanism of action of cholera toxin & other toxins. *The Indian Journal of Medical Research*.

[121] Ikigai H., Toda M., Okubo S., Hara Y., Shimamura T. (1990). Relationship between the anti-hemolysin activity and the structure of catechins and theaflavins. *Japanese Journal of Bacteriology*.

[122] Toda M., Okubo S., Ikigai H., Shimamura T. (1990). Antibacterial and anti-hemolysin activities of tea catechins and their structural relatives. *Japanese journal of bacteriology*.

[123] Fukai K., Ishigami T., Hara Y. (1991). Antibacterial activity of tea polyphenols against phytopathogenic bacteria. *Agricultural and Biological Chemistry*.

[124] Horiuchi Y. O., Toda M. A., Okubo S. A., Hara Y. U., Shimamura T. A. (1992). Protective activity of tea and catechins against Bordetella pertussis. Kansenshogaku zasshi. *The Journal of the Japanese Association for Infectious Diseases*.

[125] Friedman M., Henika P. R., Levin C. E., Mandrell R. E., Kozukue N. (2006). Antimicrobial activities of tea catechins and theaflavins and tea extracts against Bacillus cereus. *Journal of Food Protection*.

[126] Hamilton-Miller J. (1995). Antimicrobial properties of tea (*Camellia sinensis* L.). *Antimicrobial Agents and Chemotherapy*.

[127] Chen C.-N., Lin C. P. C., Huang K. K. (2005). Inhibition of SARS-CoV 3C-like Protease Activity by Theaflavin-3,3′-digallate (TF3). *Evidence-based Complementary and Alternative Medicine*.

[128] Yang J., Li L., Jin H. (2012). Vaginal gel formulation based on theaflavin derivatives as a microbicide to prevent HIV sexual transmission. *AIDS Research and Human Retroviruses*.

[129] Bartenschlager R., Lohmann V., Penin F. (2013). The molecular and structural basis of advanced antiviral therapy for hepatitis C virus infection. *Nature Reviews Microbiology*.

[130] Jacobson I. M., Davis G. L., el–Serag H., Negro F., Trépo C. (2010). Prevalence and challenges of liver diseases in patients with chronic hepatitis C virus infection. *Clinical Gastroenterology and Hepatology*.

[131] Chowdhury P., Sahuc M. E., Rouillé Y. (2018). Theaflavins, polyphenols of black tea, inhibit entry of hepatitis C virus in cell culture. *PLoS One*.

[132] Colpitts C. C., Baumert T. F. (2016). Hepatitis C virus cell entry: a target for novel antiviral strategies to address limitations of direct acting antivirals. *Hepatology International*.

[133] de Oliveira A., Prince D., Lo C. Y., Lee L. H., Chu T. C. (2015). Antiviral activity of theaflavin digallate against herpes simplex virus type 1. *Antiviral Research*.

[134] Archana S., Abraham J. (2011). Comparative analysis of antimicrobial activity of leaf extracts from fresh green tea, commercial green tea and black tea on pathogens. *Journal of Applied Pharmaceutical Science*.

[135] Jang M., Park Y. I., Cha Y. E. (2020). Tea Polyphenols EGCG and Theaflavin Inhibit the Activity of SARS-CoV-2 3CL- Protease In Vitro. *Evidence-based Complementary and Alternative Medicine*.

[136] Mhatre S., Srivastava T., Naik S., Patravale V. (2021). Antiviral activity of green tea and black tea polyphenols in prophylaxis and treatment of COVID-19: a review. *Phytomedicine*.

[137] Xie Y., Xiao J., Fu C., Zhang Z., Ye Z., Zhang X. (2018). Ischemic preconditioning promotes autophagy and alleviates renal ischemia/reperfusion injury. *BioMed Research International*.

[138] Venkatachalam M. A., Weinberg J. M., Kriz W., Bidani A. K. (2015). Failed tubule recovery, AKI-CKD transition, and kidney disease progression. *Journal of the American Society of Nephrology*.

[139] Nisar M. F., He J., Ahmed A., Yang Y., Li M., Wan C. (2018). Chemical components and biological activities of the genus phyllanthus: a review of the recent literature. *Molecules*.

[140] Thiele J. R., Zeller J., Kiefer J. (2018). A conformational change in C-reactive protein enhances leukocyte recruitment and reactive oxygen species generation in ischemia/reperfusion injury. *Frontiers in Immunology*.

[141] Shao L., Luo Y., Zhou D. (2014). Hematopoietic stem cell injury induced by ionizing radiation. *Antioxidants & Redox Signaling*.

[142] Balaban R., Nemoto S., Finkel T. (2005). Mitochondria, oxidants, and aging. *Cell*.

[143] Wang L., Tu X. H., Zhao P., Song J. X., Zou Z. D. (2012). Protective effect of transplanted bone marrow-derived mesenchymal stem cells on pancreatitis-associated lung injury in rats. *Molecular Medicine Reports*.

[144] Li Z., Zhu J., Wan Z., Li G., Chen L., Guo Y. (2021). Theaflavin ameliorates renal ischemia/reperfusion injury by activating the Nrf2 signalling pathway _in vivo_ and _in vitro_. *Biomedicine & Pharmacotherapy*.

[145] Wang X. (2001). The expanding role of mitochondria in apoptosis. *Genes & Development*.

[146] Farkhondeh T., Folgado S. L., Pourbagher-Shahri A. M., Ashrafizadeh M., Samarghandian S. (2020). The therapeutic effect of resveratrol: focusing on the Nrf2 signaling pathway. *Biomedicine & Pharmacotherapy*.

[147] Diao C., Chen Z., Qiu T. (2019). Inhibition of PRMT5 Attenuates Oxidative Stress-Induced Pyroptosis via Activation of the Nrf2/HO-1 Signal Pathway in a Mouse Model of Renal Ischemia- Reperfusion Injury. *Oxidative Medicine and Cellular Longevity*.

[148] Abd El-Megeid A. A., IZ A. A., Elsadek M. F., Abd El-Moneim Y. F. (2009). The protective effect of the fortified bread with green tea against chronic renal failure induced by excessive dietary arginine in male albino rats. *World Journal of Dairy & Food Sciences*.

[149] Imran A., Arshad M. U., Arshad M. S., Imran M., Saeed F., Sohaib M. (2018). Lipid peroxidation diminishing perspective of isolated theaflavins and thearubigins from black tea in arginine induced renal malfunctional rats. *Lipids in Health and Disease*.

[150] Kaur S., Greaves P., Cooke D. N. (2007). Breast cancer prevention by green tea catechins and black tea theaflavins in the C3 (1) SV40 T, t antigen transgenic mouse model is accompanied by increased apoptosis and a decrease in oxidative DNA adducts. *Journal of Agricultural and Food Chemistry*.

[151] Ukil A., Maity S., Das P. K. (2006). Protection from experimental colitis by theaflavin-3, 3′-digallate correlates with inhibition of IKK and NF-*κ*B activation. *British Journal of Pharmacology*.

[152] Sajilata M., Bajaj P. R., Singhal R. (2008). Tea polyphenols as nutraceuticals. *Comprehensive Reviews in Food Science and Food Safety*.

[153] Maity R., Chatterjee M., Banerjee A. (2019). Gold nanoparticle-assisted enhancement in the anti-cancer properties of theaflavin against human ovarian cancer cells. *Materials Science and Engineering: C*.

[154] Ding Y., Zou L., Lu C., Tong H., Chen B. (2018). In situenzymatic synthesis and purification of theaflavin-3,3′-digallate monomer and incorporation into nanoliposome. *International Journal of Food Science & Technology*.

[155] Jiang Y. (2017). *Novel polysaccharide-polypeptides nanocomplexes: assembly, characterization, and applications in delivery of black tea polyphenols*.

[156] Shutava T. G., Balkundi S. S., Vangala P. (2009). Layer-by-layer-coated gelatin nanoparticles as a vehicle for delivery of natural polyphenols. *ACS Nano*.

[157] Hammond S. J. (2015). *Formation of Enriched Black Tea Extract Loaded Chitosan Nanoparticles via Electrospraying*.

[158] Kulandaivelu K., Mandal A. K. A. (2017). Improved bioavailability and pharmacokinetics of tea polyphenols by encapsulation into gelatin nanoparticles. *IET Nanobiotechnology*.

[159] Liu C., Zhang Z., Kong Q., Zhang R., Yang X. (2019). Enhancing the antitumor activity of tea polyphenols encapsulated in biodegradable nanogels by macromolecular self-assembly. *RSC Advances*.

[160] Shao P., Zhang H., Niu B., Jin W. (2018). Physical stabilities of taro starch nanoparticles stabilized Pickering emulsions and the potential application of encapsulated tea polyphenols. *International Journal of Biological Macromolecules*.

